# Construction of Interactive Virtual Reality Simulation Digital Media System Based on Cross-Media Resources

**DOI:** 10.1155/2022/6419128

**Published:** 2022-08-05

**Authors:** Shuo Li, Jianjun Li

**Affiliations:** ^1^The Arts Faculty of North University of China, Taiyuan, China; ^2^Xishan Coal and Electricity Group Co., Ltd., Taiyuan, China

## Abstract

The combination of video and music is the most typical combination form in interactive multimedia works, which focuses on the audio-visual presentation characteristics of interactive art. Since both creative practice and theoretical research are still in the development stage, we focus on the creation of audio-visual integration in interactive multimedia works. Theoretical achievements are still very rare, and the guidance of creation theory plays an important role in the improvement of the aesthetic level of works. Therefore, for the development of interactive multimedia works creation, creating a new audio-visual relationship research path has important theoretical value and application value. It also has a certain historical significance for promoting the maturity of this art form. Through interactive virtual reality technology, this paper conducts an in-depth discussion on the simulation of digital media system across media resources. It is more suitable for the user's preference than the PC machine side. From technical means to artistic aesthetic characteristics and practical application, the application field and industry influence of digital media art carried by virtual reality are expounded, and the problems and solutions faced at this stage are proposed. By analyzing the application of virtual reality aesthetics in interaction design, the relationship between the visual level and the experience level of virtual reality aesthetics is discussed. Starting from the basic concepts of virtual reality aesthetics and interaction design, this paper analyzes the virtual reality space architecture and aesthetic dimension of interaction design in the era of artificial intelligence, and the value of virtual reality aesthetics in interaction design. Most interactive multimedia works rely on the open programming environment and have highly open creation tools to realize cross-media creation. The interactive integration of multimedia art and visual communication is the trend in design development. It follows the law of formal beauty and uses visual language to guide the content. Visual communication adapts to the needs of multiplatform media communication, adds multimedia art elements, and promotes the integration of scientific and technological progress and artistic development.

## 1. Introduction

After collecting information from multiple channels, an interactive “wall free” environment and a user action information simulation system are generated. Users can enter a virtual reality environment in such a simulation system, immerse themselves in a series of intuitive sensory sensations in the virtual world, actively and passively connect with the system through their responses, and extend their behavioural attributes to the virtual direction [1]. First, the operation interface of the mobile terminal can present a combination of virtual and real scenes on the full screen, which further increases the audience's sense of immersion and presence. At present, the virtual reality industry at home and abroad is characterized by huge investments stimulating the rapid development of industry chain links, gradually moving from the diverse consumer side of each layer to industry applications. Due to the gradual enrichment of virtual reality “drawing” content and the increasing experience satisfaction of immersive roaming communities, the revenue tendency of relying entirely on the built-in level of hardware devices has changed at the right time, making online transactions of leisure services the leading form of consumption. Coupled with the development of a virtuous cycle of hardware R&D revenue itself, the enrichment of virtual reality creative content and the promotion of the creative economy accelerate the development of the virtual reality industry. The combination of virtual reality and other traditional industries has more kinds of potential that can be encouraged and opportunities that can be strived for.

The rapid development and update of virtual reality technology have made its potential to replace the existing PC as the new generation of computing platforms gradually revealed, while the depth and breadth of its application in other traditional industries are also expanding. The immersive and interactive experience that virtual reality technology can provide to users is often missing, but it is urgently needed in other traditional industries, which is the reason for the emergence of the concept of “virtual reality+.” With the development of digital technology, humankind has entered a new “digital media” information dissemination society. Along with this platform of digital media, digital media art has emerged, and its vitality and development prospects are huge and immeasurable [2]. As a diversified new art field, digital media art is also firmly branded with “technology,” and the emergence of virtual reality technology brings a brand-new stage for digital media art. It is believed that the continuous integration with virtual reality technology will provide a boost to the development of more industries. Immersion means that the user can be surrounded by the virtual environment and the realism of the virtual environment is reinforced by various feedback. Based on human physiological and psychological characteristics, virtual reality technology generates realistic three-dimensional graphics from the computational rendering layer and then provides users with a variety of natural interactions and feedback through the interaction layer to achieve extraordinary immersion [3]. Compared to other computing platforms, the immersion effect is one of the most important indicators of virtual reality, and the user's sense of presence tests the performance of virtual reality devices.

Virtual reality news documentaries mostly focus on more realistic topics, which is an innovation in the context of virtual reality technology applied in news communication. The intervention of virtual reality technology reshapes the production of news documentaries, following the principle of content authenticity of news documentaries, and increases the interactive role that distinguishes from 360-degree panoramic video news. It can provide a reference standard for the redirection algorithm, thereby helping to propose a better redirection algorithm. The reality of virtual reality is a reality built on human perception, experiencing the user as a measuring tool. The virtual art of expression allows for further enrichment of the animated presentation of news documentaries. Virtual reality technology does not affect the true artistic nature of news documentaries, whether it is the simulation of scientific experiments, the need to restore historical originality, the need for specialization of artistic expression, or in the communication exhibition of education, the content and theme presented by them can be visually reconciled with the help of virtual reality technology [4]. As an auxiliary technical means, news documentaries adhere to the bottom line of the authenticity of the creative content and achieve the artistic interlacing effect, that is, users can more intuitively and easily identify the artistic expression effect brought by virtual reality technology and will not fall into the misunderstanding and experience of confusing animation technology and documentary filming. At the same time, the artistic interstitial effect follows the bottom line and ethical requirements of news documentary creation, for news documentaries to reach a higher level of art and constantly improve, expand the aesthetic needs of the audience, inspire users to think about their sense of identity and society, not only enrich the technical and artistic creation methods of news documentaries but also use virtual reality technology to map the humanistic and aesthetic space, awaken the emotional world inside users, and generate diversity of resonance and new senses, thus enabling users to truly express their audio-visual thinking.

## 2. Related Works

Digitalization has become an extension of people's perception of the world and a new tool to change it, playing a major role in the development of contemporary society and thus influencing its place in the creation of visual arts [5]. The redirection algorithm based on an artificial potential energy field can provide a theoretical basis for the specific value of redirection gain by analyzing the resultant force from the real scene tracking area or the virtual scene received by the user. Because of its immense applications in training and testing, virtual reality technology is often used first in sectors such as defense and aerospace and then gradually spread to industries such as healthcare, education, and entertainment, which have developed huge sales markets for it and reaped lucrative economic benefits [6]. In just a few decades, virtual reality technology has become increasingly perfected for every aspect of everyone's daily life, making it possible for managers, leaders, and engineers to use, modify, and design the designed systems operationally in a virtual reality environment to make them better [7]. By conducting military exercises in a virtual scenario, it seems that everything is in the actual exercise process and trained military personnel can feel the feeling of being surrounded. This simulated scene has a strong sense of reality, which will make the experimenter feel pain, which is conducive to the transition from virtual scene to real battlefield environment, which for the military activities will be a long-term and far-reaching impact [8].

In it, we propose a method for measuring the perceptual quality of the 360-degree panoramic video, that is, a comparative study by experimentally comparing the peak signal-to-noise ratio of the ordinary video and processed video in the original test sequence sample during the user's field of view in a flat view experience [9]. This method considers the actual visual threshold of the user during the experience and indirectly validates a better evaluation method [10]. However, these evaluation models only focus on the study of perceptual quality measurement of 360-degree panoramic video and have not yet considered the real sense of virtual reality news video under the redefinition and classification of this study [11]. Especially in recent studies, there is a single lack of research content and research methods for user perception quality assessment measurement of news documentaries under virtual reality mobile development [12]. User experience is the user's comprehensive consideration of the communication quality of that especially emerging media, and the user's perceived quality is directly related to the application characteristics of the digital media to be measured, and in the virtual world, there are others such as the sense of immediacy [13]. Therefore, the assessment of the perceived quality of digital media users needs to focus not only on the performance and quality parameters of hardware devices but also on the measurement and assessment of the quality of user experience considering proprietary differences.

It is considered that packaging can use the concept of virtual reality in the design of structure and decoration. The use of virtual space can make the packaging structure rich and interesting. From the function of modern product packaging design, attention should be paid to the use of virtual space in packaging design to maximize its use to a certain extent; and virtual reality design in packaging and decoration focuses on three aspects: packaging fonts, packaging colours, and packaging graphics. There is a dialectical relationship between the publicity and individuality produced by new media art, which are both different from each other and connected with each other. Designers make full use of virtual and three-dimensional methods to create the aesthetic method of “virtual reality” to enhance the visual impact of graphics and stimulate the imagination of the audience design models. There are many similar methods and means of virtual design through graphical or decorative graphic language on the market today, which allows consumers to understand the product briefly by contrasting it with the virtual space around other design elements. We can also enhance the attractiveness of the images by creating a “bottom-up” approach.

## 3. Interactive Virtual Reality Simulation Analysis

Virtual reality was first used in NASA and the military to stimulate scientific research and testing. It works by using a computer graphics generator to generate a simulated realistic scene: a position tracker to determine the actual orientation and trajectory of the object in the virtual space and, finally, a multifunctional sensor controller to realize the control of the virtual scene by the participants, bringing them an immersive sense of immersion [14]. To better improve the realism and immersion of the virtual reality simulation system, virtual humans need to be added to the VR system as a substitute for real people in the VR environment. With the continuous development trend of virtual reality technology, avatars have an increasingly important role in VR systems. In terms of virtual human research, virtual human 3D modelling technology and virtual human motion control technology are the most concerned in the industry. In the new media environment, the most prominent form of art is virtual reality art. Virtual reality also includes many disciplines.

The VR system architecture mainly consists of three parts: foundation layer, support layer, and application layer. The foundation layer provides the underlying hardware support, including Qualisys optical motion capture hardware system, computer server, network communication, HTC VIVE headset hardware system, and so on; the support layer uses mature commercial software to provide virtual human motion driver, scene simulation, motion data acquisition, and so on; and the application layer is supported by the corresponding software, through integration and secondary development, to realize the VR scene construction, virtual human loading VR scene, data acquisition, data conversion, and driving virtual human motion and other functions. The architecture of the motion-capture-based VR system is shown in Figure 1.

The software part is mainly TQM software, which is mainly used to display the spatial location of the marker points, and the motion capture software facilitates the user to display and operate the marker points in 3D; the hardware part is mainly used to collect the position information of the marker points on the human rights [15]. The most prominent feature of virtual reality technology is the authenticity of human sensory feedback. Virtual reality technology not only leads the technology of the times trend. The server runs Unity 3D software to display the scene and load the avatar and connects to the motion capture server to obtain the collected data through the interface developed for Unity 3D. The server transforms the acquired marker point data information through the interface function and then uses the transformed joint translation angle to immediately drive the virtual human rigid body movement to execute the actions made by the motion capture model (the volunteer used to collect data in the motion capture area).

(1) $$\begin{array}{c} F_{S}=C\frac{d}{\left\|d^{2}\right\|}\times \frac{1}{d^{\lambda }}. \end{array}$$

There are a variety of scenarios for the use of virtual reality inside the range of mobile applications. It is favoured by most users because of the mass and convenience of mobile. Developers generally choose to develop mobile applications because the overlapping realistic effect of virtual reality applications on mobile is more suitable for users' preferences than PC machines. First, the mobile interface can present a full-screen combination of virtual and real scenes, which increases the viewers' immersion and sense of presence; secondly, the mobile terminal can use the rear camera of the cell phone to capture the relevant features of the actual interface in front of the lens and import it to the app at the same time, which can better show the viewers the combination of virtual and real scenes and adopt the dual-camera mode at the same time. The final point is in the field of interaction design profitability so that customers can use gestures directly without the limitations of interactive devices, optimizing the natural experience of interaction.

(2) $$\begin{array}{c} F_{b}=\sum_{i=1}^{n}ke_{i}^{2}\times \frac{1}{d_{\lambda }^{i}}. \end{array}$$

In addition to using the geometric nature of the tracking area, it is also possible to determine one or more safety points in the tracking area according to the researcher's or user's own needs, but the safety points must meet the three conditions mentioned above, and when there are multiple safety points, the gravitational force of multiple safety points can be calculated separately, but in the final calculation of the combined force of the tracking area, only the gravitational force of one of the safety points can be selected for the combined force. The final calculation of the combined force in the tracking area can only be done by selecting one of the safety points. For convenience, the geometric centre of the tracking area is used as the only safety point in the following equation:

(3) $$\begin{array}{c} F_{\text{VGi}}=V\frac{d}{\left\|d^{2}\right\|}\times \frac{1}{d^{\alpha }}P_{i}^{2}. \end{array}$$

As the field of architecture continues to be explored, new research questions arise on how to apply the questions and reflections obtained from postuse evaluations to architectural design. The purpose of this section is to demonstrate that the introduction of the concept of artificial potential field in the redirection algorithm can provide a reference standard for the redirection algorithm and thus contribute to the formulation of better redirection algorithms. First, we consider the connection between traditional redirection algorithms and artificial potential field redirection algorithms [16]. The online and offline cross-media dissemination of scientific information can help users recognize and understand innovative science and technology and provide an effective way to popularize scientific information to the public. The core idea of the S2C algorithm is to guide the user's movement path through the centre of the tracking region. Therefore, it can be regarded as an artificial potential field redirection algorithm with the safety point as the geometric centre of the tracking region and without considering the tracking region repulsion and virtual scene cohesion. If the safety point is artificially increased on this basis, again without considering other conditions, the schematic diagram of the multicentre point guidance algorithm is shown in Figure 2.

Next, consider the connection between the traditional reset algorithm and the artificial potential field-based reset algorithm proposed in this paper. The principle of the freeze steering algorithm is to wake up the virtual scene after freezing (suspending) the motion of the virtual scene before a collision occurs and making the user rotate by a certain angle. Therefore, it is only necessary to note down the user rotation angle and substitute it into the reset algorithm proposed in this paper. Make the leisure service online transaction a leading consumption form. Coupled with the virtuous cycle development of hardware R&D revenue itself, the enrichment of virtual reality creative content and the promotion of the creative economy accelerate the development of the virtual reality industry. Therefore, despite the different operations during the reset, the freeze steering algorithm and the reset algorithm in this paper can theoretically guide the user to the same route after the reset. Similarly, for the 2:1 steering algorithm, it is also possible for the two different algorithms to steer the user to the same path.

Some of the traditional redirection algorithms are based on a particular instance of the artificial potential field redirection algorithm. By changing the relevant parameters of the artificial potential field redirection algorithm, it is theoretically possible to overlap the user's guidance path with that of the traditional redirection algorithm. The artificial potential field-based redirection algorithm, by analyzing the combined forces that the user is subjected to from the real scene tracking area, or the virtual scene, can provide a theoretical basis for the specific value of the redirection gain, thus contributing to the proposal of a more reasonable redirection algorithm.

(4) $$\begin{array}{c} F_{v}^{2}=F_{VGj}^{3}. \end{array}$$

New media art with public nature, in the context of the world, is being impacted by the trend of information technology; through the Internet, the distance between people is getting closer and closer, so that different cultures and different living environments can be exchanged. At the same time, in the new media, individual information is unique and has diversified characteristics, and the basic characteristics of new media include sharing, interactivity, and openness, while the public and individual nature of new media art are both distinct from each other and related to each other in a dialectical relationship. In society, art itself is expressed from the life of the public, which makes the public participate in new media art activities together and feel the charm of new media art [17]. The public character of new media art makes art gradually get rid of the historical tradition of bending high and low names, which seems to be able to let only a few people participate, and can make art come into closer contact with the public and make art appreciation and art creation become a part of the public's daily life so that all people can be imbued with art atmosphere.

The construction of authenticity of news documentaries based on virtual reality technology needs more reshaping of documentary aesthetics theory. Compared with the technical problems of virtual reality news documentaries, the exploration of virtual reality news documentaries from the aesthetic perspective has more prominent theoretical and practical significance. It also brings a new stage for the display of digital media art. The traditional 2D news documentary video production process is indeed an increasingly skilled situation, but to highlight the design aesthetics of media design thinking, there are still technical shortcomings and unmet user needs, and even in the future macro view, the longer this conservative time lasts, the greater the impact of dragging the leg maybe.

### 3.1. Cross-Media Resources of Digital Simulation Media System Design

With the impact of the trend of information technology, the environment in which people live is contained by the digital industry, due to the wide range of information dissemination content, a large amount of information, and rapidly so that there is no longer any privacy between people, from the fundamental search for small changes. In this era, new media art is created. New media art and traditional art have obvious differences in both the creation method and the form of communication [18]. New media art reflects more of a fusion of technology and art; technology includes computers, video, Internet, and so on. New media art has brought different art forms, among which the most prominent is virtual reality art, and virtual reality technology especially highlights the reality of human sensory feedback. Virtual reality technology does not only lead the trend of the technology of the times but also exists in new forms of artistic expression when art and technology fuse with each other to produce works that make the experience more beautiful and more comfortable. Virtual technology and art guide and complement each other, although virtual art is mostly realized on the premise of technology, technology is like a pen. If you want to draw a good look on the screen, you need art to foil it to make it more beautiful.

Virtual reality art shows that three-dimensional space cannot be compared with traditional art, two-dimensional visual effects are not as good as three-dimensional space. People's response to space usually requires feedback from external things, that is, the division of light, line, and surface. Through a more detailed arrangement of the visual senses of the human perspective, the experiencer can better feel the three-dimensional sense of space, as shown in Figure 3.

In the virtual reality system, users can experience the five senses of objects in the virtual world through a series of sensing devices. For example, the participant sees a virtual object through the virtual reality system and at the same time can also touch the object with their hands, as in the real world in general the participant can feel the sensation of the hand touching the object, which is the haptic effect achieved by sensing feedback technology [19]. It is believed that the continuous integration with virtual reality technology will be able to aid the development of more industries. 

This practical project hopes to explore the possibilities of such science digital design through the digital presentation of two- and three-dimensional dynamic graphics while maintaining the aesthetics unique to the art and design profession and to create science digital works that are accessible to everyone, with the general user as the target audience. Studies have shown that scientific visualization through cross-border cooperation between science and art is an effective way to present innovative scientific content because of its rational scientific connotation and emotional visual aesthetics. The cross-media dissemination of scientific information online and offline can help users recognize and understand innovative science and technology, providing an effective way to popularize scientific information to the public.

The spontaneous comments reflect the diverse needs of visitors for architectural functions from the perspective of ordinary people. Dining and shopping account for 30.74% of the attention in the behaviour category, and the amount of attention for both is stable and almost independent of month-to-month changes. This indicates that service functions are an important part of the complete museum experience. At the same time, parking, which received much more attention than “public transportation,” indicates that accessibility and ease of travel are also important evaluation criteria in the development and operation of art museums.

Since a complete virtual reality system has not only real scenes but also virtual scenes. This section focuses on the ensemble algorithm of virtual scenes. Unlike the many limitations of real scenes, virtual scenes are not limited to real physical space and corresponding hardware technology (e.g., current hardware technology limits the size of the tracking area but cannot limit the size of virtual scenes). The construction of virtual scenes depends to a large extent on the wishes of the virtual reality system developers [20]. The intervention of virtual reality technology has reshaped the production of news documentaries, followed the principle of content authenticity of news documentaries, and increased the interaction that is different from 360-degree panoramic video news. Therefore, it can be said that virtual scenes are free at this stage. Nevertheless, for the sake of simplifying the problem, the virtual scenes targeted in this paper are only oriented to simple flat scenes, that is, scenes without height variation or with only simple height variation. The scenes with simple height changes are like “floors” that can be considered as multiple independent planar scenes, which are connected by simple passages (stairs), as shown in Figure 4.

To verify the effectiveness of the virtual scene cohesion, two control groups are set up for comparison. The first group is the no redirection group without using any gain; the second group is the redirection group using the virtual scene ensemble force proposed in this paper. In this paper, different gravitation is used according to the current state of the user. In this paper, we detect the user's grasping state to determine the user's current state. When the user does not grasp any object, we detect the directional vector angle between the front of the user's field of view and the position of all objects pointing from the user's position to the “active” state, and the object with the smallest angle exerts a gravitational force on the user, and the redirection gain is used to guide the user to the object. When the user grabs an object, the target area corresponding to the object exerts a gravitational force on the user, and the redirection gain is used to guide the user to the target area. When the object is placed in the target area, the object is “inactive.”

## 4. Results and Analysis

### 4.1. Performance Analysis of the Interactive Virtual Reality Simulation System

The results were statistically analyzed using SPSS software, and the normality was calculated using the Kolmogorov–Smirnov test. In this section, we assessed the significance of throwing accuracy by several factors, including the environment in which the participants were located, the target walking trajectory (3: vertical, straight, and circular) and the target walking speed, and the distance (2:4.6 m and 6.7 m, i.e., the distance from the free-throw line and the distance from the three-point line of the basketball court, respectively). In addition, a multifactor ANOVA was performed on the collected data. Throwing experiments were executed in both virtual and real environments, and all factor combinations are shown in Figure 5.

At 4.6 m, the average throwing accuracy is 51.9% in VR and 68.2% in the real scene, which is 31.4% higher than in VR; at 6.7 m, the average throwing accuracy is 41.4% in VR and 46.0% in the real scene, which is 11.1% higher than in VR. In VR and the real world, other factors are the same, the greater the distance, the lower the accuracy; on the other hand, the greater the distance between VR and the real scene, the smaller the gap becomes apparent. According to Figure 5, these observations can be verified in the walking “trajectory” factor. Moreover, this factor has a significant factor of *P* < 0.01 in VR and *P* < 0.01 in the real world, which means that the ‘distance' factor is more dominant in the real-world environment. Whether it is in the simulation of the effect of scientific experiments, the need to restore the original appearance of history, the need for special artistic expression effects, or the communication and expansion of the importance of educational significance, the content and themes presented can be visualized with the help of virtual reality technology.

The average throwing accuracy was 48.8% in VR and 76.0% in the real-world scenario with the target “static,” which was 55.7% higher than in VR; the average throwing accuracy was 46.7% in VR and 58.7% in the real-world scenario with the target walking at a “uniform” speed. The average throwing accuracy was 46.7% in VR and 55.7% in the real scene, which was 19.3% higher than that in VR; the average throwing accuracy was 46.7% in VR and 55.7% in the real scene when the target walked at “variable speed.”

In the real environment, the throwing accuracy decreases as the target walks at a different speed and further decreases if the target moves at a variable speed. However, in the virtual environment, the throwing accuracy remains almost unchanged regardless of the target's walking speed. We obtained this observation because the significant factor is *P* > 0.05 in VR and *P* < 0.001 in the real world, which means that the walking “speed” factor is dominant in the real world but has no effect in VR.

The greater the distance, the smaller the gap between VR and real-world scenes. These observations are further confirmed by the data in Figure 6, where the “constant” and “random” elements are very small because they have different walking trajectories and different distances. Based on these observations, we believe that the participants' performance in VR was dependent on their skills with the VR device rather than their original skills and knowledge of basketball in the real world.

When the target walked in a “straight” line, the average throwing accuracy was 56.7% in VR and 64.8% in the real scenario, which is 14.3% higher than in VR; when the target walked in a “vertical” line, the average throwing accuracy was 42.0% in VR and 42.0% in the real scenario. When the target walks in a “vertical” trajectory, the average throw accuracy is 42.0% in VR and 52.0% in real scenes, which is 23.8% higher than that in VR; when the target moves along a “circular” trajectory, the average throw accuracy is 41.3% in VR and 54.4% in real scenes, which is 31.7% higher than that in VR. To continuously improve news documentaries to a higher artistic level, expand the audience's aesthetic needs, stimulate users' thinking about their own sense of identity and social sense, and not only enrich the technology and artistic creation methods of news documentaries. First, when the target walks back and forth in a “straight line,” the target's vision is relatively stationary, so its accuracy is higher compared to other trajectories. With these observations, the results of the experimental analysis reaffirm that the throwing accuracy of “static” targets is higher than that of “moving” targets, which is consistent in both VR and the real world. Furthermore, the significant factor of this factor is *P* < 0.001 in VR and *P* < 0.005 in the real world, indicating that the “trajectory” factor is more dominant in the virtual environment.

Finally, the overall average throwing accuracy was 47.0% in the VR scenario and 59.8% in the real-world scenario, with a significant factor of *P* < 0.001, but the participants' performance was significantly higher in the real-world environment than in the virtual environment by 27.2%. The performance in the 6.7 m, variable speed, circular “scenario, was more stable in both the real world and in VR. In contrast, performance was least stable in VR at 4.6 m, constant speed, circular,” and “in the real world at 6.7 m, constant speed, vertical.” The difference in average throwing accuracy between participants with/without discomfort in VR was 8.1%, compared to 3.2% in the real world. Thus, although we allowed for breaks in the VR experiment, discomfort from the VR device still resulted in a large decrease in accuracy in the virtual environment. Bring participants an immersive sense of immersion.

## 5. Analysis of Numerical Simulation Results

In past research, it has been suggested that the average positive affective score for a normal population is 29.7 and the average effective score is 14.8. The good reliability and construct validity of the PANAS have been demonstrated in previous application studies for all countries, and the age range includes adolescents and adults over the age of 13 years. In practice, some items are modified or replaced according to the wording and degree of comparison. The so-called virtual reality integration programs are experiential, and the game experience is also a popular method of experiencing virtual reality. The joint experience of body and spirit can play the role of multiple feelings and deepen cognition. This new type of physical and mental experience can be more profound and leave the audience with a different experience. The experiential nature that virtual reality technology can demonstrate is mainly composed of multiorgan perception and emotional resonance of the audience.

Artistic aesthetics plays a decisive role in virtual roaming design. For simple artistic aesthetics, beauty is revealed through the feelings of the human heart and occurs based on artistic media, just like the appreciation of watching artworks, if the viewer does not feel it through his heart, he cannot have aesthetic resonance. In the virtual roaming design of the art of aesthetics refers to the technology of communication, in the virtual space to see the things brought about by feelings, virtual space is a kind of art medium, in the space to appreciate their own emotions at will and produce aesthetic value. Just as the appreciators are experiencing the pleasure of immersion and interaction brought by virtual art, from the simplest viewing to direct feelings, the aesthetic value of art brought by virtual reality art is much higher than that of traditional art forms, as shown in Figure 7.

Visitors generally do not pay attention to the courtyard that appears on one side of the traffic space alone; when the left and right sides of the traffic space are connected to the courtyard, the two courtyards receive significantly more attention. To better improve the realism and immersion of the virtual reality simulation system, it is necessary to add virtual people to the VR system as a substitute for real people in the VR environment. In the subjective records, some experimenters temporarily abandoned the exhibition and explored the courtyard content first. Therefore, the connection of sightlines and flow lines between courtyards can effectively increase visitors' attention to them, but improper handling will disrupt the original flow line design and gallery narrative logic.

However, the systematic signage in transportation buildings cannot be directly applied to art museums. By setting up obvious signage, it can effectively improve the recognition of the local space. Therefore, such design elements at specific nodes can guide visitors with visual focal points and help them establish a sense of direction in the museum.

In this paper, 50 steering experiments were conducted, 25 of which did not use any redirection gain and 5 of which used redirection rotation gain based on virtual scene cohesion. The data relating to the time required to complete the whole experiment and the change of the user's visual field angle recorded in this experiment are compared, as shown in Figure 8, where NR denotes the control group without reorientation gain and VR denotes the experimental group with virtual scene cohesion-based reorientation. T1 denotes the time taken to grab the first object and put it into the corresponding area; T2 denotes the time taken to grab the second object and put it into the corresponding area; and TT denotes the total time taken from the beginning to the end of the experiment.

Analyzing the data, we can see that the proposed directional rotation gain based on the virtual scene ensemble can effectively reduce the angle that the user turns in the real environment when the headline of sight is rotated and slightly reduce the time spent on head rotation compared with that without any directional gain. Therefore, it can be said that the reorientation rotation gain based on the virtual scene ensemble force proposed in this paper is practical and effective.

## 6. Conclusion

In the virtual environment, the user's physical and emotional sensations are superlative to those of the real world, as if they were already expressed in the user's body rather than the artistic sensations brought about by the virtual scene. When an artist creates a work, the process and idea of creation are all included in the virtual. In art appreciation, the activities and feelings that the viewer feels and experiences are also different. In this paper, we take the interaction between virtual design and art as a new research direction, and the participation of the experiencer becomes part of the completion of the work. The motion capture software facilitates the three-dimensional display and operation of the marked points; the hardware part is mainly used to collect the position information of the marked points on the human body tights. While traditional artworks evolve from the artist's inspiration and thinking into a physical image, today's virtual art redefines the concept of art, requiring not only the artist's creative process but also the process of appreciation by the viewer, so that the form can be considered a complete work in the true sense of the word. Interactive artworks are the user and human-machine information interaction to obtain the perfect meaning. Virtual reality art design works give the experiencer an immersive feeling and increase the emotional attitude and aesthetic tendency of real social life. The future interactive art of virtual reality technology will have many products with the support of technology; the relationship between human and computer will not be limited to the present, but a more natural and harmonious form of interaction, and further break the gap between virtual and reality, so that virtual and reality can be integrated.

## Figures and Tables

**Figure 1:** Interactive virtual reality simulation system.

**Figure 2:** System modelling framework.

**Figure 3:** Month word frequency comparison.

**Figure 4:** Flow chart of steering experiment.

**Figure 5:** Throwing accuracy in the virtual (a) and real (b) environments.

**Figure 6:** Standard deviation of throwing accuracy for different combinations of factors: (a) VR, (b) random, (c) circle, and (d) straight.

**Figure 7:** The sense of direction and viewing habits of the sample group.

**Figure 8:** User's view trajectory after applying redirection gain.

## Data Availability

The data used to support the findings of this study are available from the corresponding author upon request.
